# Integrated Analysis and Validation of Autophagy-Related Genes and Immune Infiltration in Acute Myocardial Infarction

**DOI:** 10.1155/2022/3851551

**Published:** 2022-10-04

**Authors:** Yan Ding, Feng Wang, Yousheng Guo, Mingwei Yang, Huanji Zhang

**Affiliations:** ^1^Department of Cardiology, The Eighth Affiliated Hospital, Sun Yat-Sen University, Shenzhen 518033, China; ^2^Guangdong Innovative Engineering and Technology Research Center for Assisted Circulation, Shenzhen 518033, China

## Abstract

**Background:**

Acute myocardial infarction (AMI) is one of the most critical conditions of coronary heart disease with many uncertainties regarding reduction of ischemia/reperfusion injury, medical treatment strategies, and other aspects. The inflammatory immune response has a bidirectional regulatory role in AMI and plays an essential role in myocardial remodeling after AMI. The purpose of our research was tantamount to explore possible mechanisms of AMI and to analyze the relationship with the immune microenvironment.

**Methods:**

We firstly analyzed the expression profile of GSE61144 and HADb to identify differentially expressed autophagy-related genes (DEARGs). Then, we performed GO, functional enrichment analysis, and constructed PPI network by Metascape. A lncRNA-miRNA-mRNA ceRNA network was built, and hub genes were extracted by Cytoscape. After that, we used CIBERSORT algorithm to estimate the proportion of immunocytes, followed by correlation analysis to find relationships between hub DEARGs and immunocyte subsets. Finally, we verified those hub genes in another dataset and cellular experiments qPCR.

**Results:**

Compared with controls, we identified 44 DEARGs and then filtered the genes of MCODE by constructing PPI network for further analysis. A total of 45 lncRNAs, 24 miRNAs, 19 mRNAs, 162 lncRNA-miRNA pairs, and 37 mRNA-miRNA pairs were used to construct a ceRNA network, and 4 hub DEARGs (BCL2, MAPK1, RAF1, and PRKAR1A) were extracted. We then estimated 5 classes of immunocytes that differed between AMI and controls. According to the results of correlation analysis, these 4 hub DEARGs may play modulatory effects in immune infiltrating cells, notably in CD8^+^ T cells and neutrophils. Finally, the same results were verified in GSE60993 and qPCR experiments.

**Conclusion:**

Our findings suggest that those hub DEARGs (BCL2, MAPK1, RAF1, and PRKAR1A) and immunocytes probably play functions in the progression of AMI, providing potential diagnostic markers and new perspectives for treatment of AMI.

## 1. Introduction

Acute myocardial infarction (AMI) is clinically defined as cardiomyocyte necrosis consistent with acute myocardial ischemia [1, 2]. Principal current treatments for AMI include reperfusion therapy, antithrombotic therapy, anti-ischemic therapy, and other pharmacological treatments, and secondary prevention [1, 2]. AMI is one of the most unfavorable conditions in coronary heart disease (CHD), which not only impairs health and causes disability and death in CHD [3], but also imposes a heavy economic burden on society [4]. Worldwide, ischemic heart disease is now the most widespread reason for death, and its incidence is increasing [2]. Despite the tremendous progress in the detection and treatment of AMI in recent decades and the decrease in mortality with the available means of treatment, the mortality rate is still high. There are still many areas of uncertainty in terms of reduction of ischaemia/reperfusion (I/R) injury, medical treatment strategies, long-term management, need for observational data, real-world evidence, and pragmatic real-life clinical trials [1, 2].

Autophagy is the major intracellular degradation system. Cytoplasmic material is delivered to and degraded in lysosomes through autophagy. Autophagy has a vital function in sustaining the homeostatic balance in cells and organisms [5]. Studies have confirmed that dysregulation of cellular autophagy is relevant to the progression of various diseases [6–8], for instance, neurodegenerative diseases like parkinsonism, malignant tumors like breast, ovarian, colorectal, and lung cancers, cardiovascular disease like myocardial infarction, various types of cardiomyopathy, and atherosclerosis. Initially, it was shown that autophagy facilitated cell survival [9]; however, it was also later determined to be involved in cell death [10]. Prolonged and excessive autophagy might contribute to cell death [11]. It is generally agreed that adaptively induced autophagy or baseline autophagy contributes to the reduction of ischemia or ischemia/reperfusion injury in AMI, whereas excessive autophagy is detrimental [12].

Immune cells are involved in or associated with the immune response and include monocytes/macrophages, neutrophils, lymphocytes, and dendritic cells. It has been shown that immune cell infiltration is implicated in the development of a great many diseases like tumors [13], central system diseases [14], and skin diseases [15]. Various kinds of immune cells play diverse roles during the development of AMI [16, 17]. As the molecular mechanisms behind cellular autophagy and the immune system are better understood, the tight relationship of them is slowly being uncovered [18]. And numerous studies have shown that autophagy-mediated modulation of the immune system may enhance or diminish the effects of immunotherapy, with the potential for future use in the treatment of a wider variety of tumors [19]. In addition, with the development of sequencing technologies and genomics [20, 21] and the development of gene-related predictive tools based on disease databases [22], they can be used to provide predictive value for the risk prognosis of diseases with potential benefits for patients. However, an integrated analysis of autophagy and immunity in the pathogenesis and development of AMI has not been reported.

In our research, we identified autophagy-related hub genes by searching for DEARGs in AMI and constructed PPI network and lncRNA-miRNA-mRNA ceRNA network. Then, we compared the immune cell composition between AMI and normal subjects by CIBERSORT algorithm analysis and co-expressed hub genes with differential immune cells. Finally, we performed a multidimensional validation at the level of another dataset and qPCR experiments of the 4 identified hub DEARGs to speculate on the underlying mechanisms of AMI development.

## 2. Materials and Methods

### 2.1. Data Selection and Analysis of Differential Gene Expression

The gene expression profiles analyzed in our research were taken from the Gene Expression Omnibus (GEO) database [23] (https://www.ncbi.nlm.nih.gov/geo/). The GEO database is an international public repository for storing microarray, second-generation sequencing, and other high-throughput sequencing data [23]. The mRNA expression profiles used for the analysis in our work were obtained from 7 AMIs (STEMI) and 10 control samples in dataset GSE61144 [24], and the miRNA expression data were obtained from 20 AMI and 64 control samples in dataset GSE31568 [25]. Differentially expressed mRNAs (DEmRNAs) or differentially expressed miRNAs (DEmiRNAs) from AMI and normal specimens were identified via GEO2R online tool [23] (https://www.ncbi.nlm.nih.gov/geo/geo2r/) with |log2 FC| > 0.5 and adj. *P* values <0.05. GEO2R is a web application based on *R* analysis that facilitates the identification and visualization of differential gene expression [23].

### 2.2. Identification of Differentially Expressed Autophagy-Related Genes (DEARGs)

The human autophagy database (HADb) is the first human autophagy-dedicated database, developed in the tumor immunotherapy and microenvironment (TIME) group at the Luxembourg Institute of Health. There are over 200 humankind genes/proteins associated with autophagy manually collected from the biomedical literature and other online resources listed [26]. We extracted all autophagy-related genes (ARGs) in HADb and then obtained 44 DEARGs after taking the intersection with DEmRNAs in GSE61144 by a Venn diagram.

### 2.3. GO/Metascape Enrichment Analysis and PPI Network Construction

Metascape [27] (https://metascape.org/gp/index.html) integrates over 40 independent data sources and is updated monthly. The pathway enrichment analysis by Metascape uses GO, KEGG, Reactome, and MSigDB. It calculates pairwise similarities between any two enriched terms based on Kappa-test score [28], automatically clusters the enriched terms into nonredundant groups, and then performs hierarchical clustering of similarity (0.3 similarity threshold) matrices. Metascape selects the most significant (lowest *P* value) term in each cluster and represents that cluster in the form of a bar chart and heat map. Metascape utilizes BioGrid's [29] protein-protein interactions as the primary data source, complemented by InWeb_IM [30] and OmniPath [31], and applies the MCODE algorithm [32] to automatically extract protein complexes embedded in the large networks and combines the three most significantly enriched ontology terms to annotate putative biological roles for each MCODE complex. We used Metascape to analyze DEARGs to reveal their gene annotation and functional enrichment and then constructed the PPI networks.

### 2.4. Construction of miRNA-lncRNA-mRNA ceRNA Regulation Network

Starbase [33] (https://starbase.sysu.edu.cn/), miRDB [34] (http://mirdb.org/), and DIANA-TarBase v.8 [35] (http://www.microrna.gr/tarbase) are used for predicting miRNAs. Starbase (https://starbase.sysu.edu.cn/), miRcode [36] (http://www.mircode.org/), and lncbase v.2 [37] (http://carolina.imis.athena-innovation.gr/diana_tools/web/index.php?r=lncbasev2/index-predicted) are used for predicting lncRNAs. StarBase v2.0 provides the most comprehensive network of miRNA-mRNA and miRNA-lncRNA interaction network supported by CLIP-Seq experiments to date [33]. MiRDB can be used for miRNA target prediction and functional annotation by employing an improved algorithm [34]. DIANA-TarBase v8 provides experimentally supported information on the regulation of miRNA-mRNA [35]. MiRcode identifies putative target sites based on seed complementarity and evolutionary conservation, and it allows putative microRNA–target sites in lncRNAs of interest or predicted targets of specific microRNAs [36]. LncBase provided a database of experimentally supported and in silico predicted miRNA Recognition Elements (MREs) on lncRNAs [37]. As a result, based on the acquired lncRNAs, miRNAs, mRNAs, and their interactions, the miRNA-lncRNA-mRNA ceRNA regulation network was constructed by Cytoscape [38].

### 2.5. CIBERSORT Estimation

For the purpose of evaluating the proportion of 22 immunocyte kinds from AMI and normal samples, we applied the CIBERSORT algorithm [39]. It was considered worthwhile for further analysis only for those specimens with a CIBERSORT output value of *P* < 0.05. For the purpose of determining potentially important immune infiltration cell subsets between the AMI and normal group, Wilcoxon rank-sum test was applied for subsequent analysis.

### 2.6. Correlation Analysis of the Autophagy-Related Genes and Immunocytes

In order to uncover the possible associations between ARGs and immune cells, Pearson correlation analysis was used to calculate the CIBERSORT algorithm output values. We analyzed the correlations between 4 hub DEARGs and 5 kinds of immune cell subpopulations from all samples.

### 2.7. Multidimensional Validation

Finally, to verify the reliability of the dataset analysis results, we performed multidimensional validation. We verified the gene expression in another GEO dataset and in human cardiomyocyte qPCR experiments. The mRNA expression profiles were taken from 7 AMI (STEMI) and 7 control specimens in dataset GSE60993 [24]. Differences with a *P* value <0.05 were deemed statistically significant. To further validate the previous results of our findings, we performed cellular experiments, cell culture, hypoxia model construction, and qRT-PCR as described following.

### 2.8. Cell Culture and Treatment

The human myocardial AC16 cell line was purchased from American Type Culture Collection (ATCC, Manassas, VA, USA) and cultured in Dulbecco's Modified Eagle's Medium (DMEM; Gibco, Grand Island, NY, USA) supplemented with 10% fetal bovine serum (FBS; Gibco, Grand Island, NY, USA), 100 U/ml penicillin and 100 *μ*g/ml streptomycin at 37°C in a humid atmosphere with 5%CO2. Cells were exposed to hypoxia conditions (94% N2, 1% O2, and 5% CO2) for 4 h, and cells incubated under normally conditions were used as control.

### 2.9. Quantitative Real-Time PCR (qRT-PCR)

The manufacturer's guide provided instructions for obtaining total RNA from AC16 cells by using TRIzol reagent (Invitrogen; Thermo Fisher Scientific, Inc., MA, USA), and we quantified RNA by measuring absorbance at 260 nm using NanoDrop ONE (Thermo Fisher Scientific, Inc., MA, USA). The Evo M-MLV RT Kit (Accurate Biology, Hunan, China) was applied to reverse transcribe RNA into complementary DNA. The qPCR was performed on Roche LightCycler 480 II (Roche Diagnostics, Mannheim, Germany) using cDNA as template. Reaction mixtures (10 *μ*l) were prepared using SYBR® Green Premix Pro Taq HS qPCR Kit II (Accurate Biology, Hunan, China), and PCR was accomplished by following the manufacturer's instructions. The internal standard was glyceraldehyde-3-phosphate dehydrogenase (GAPDH). The following primers were used: BCL2-F: 5′-AGATTGATGGGATCGTTGCCT-3′; BCL2-R: 5′-CAGTCTACTTCCTCTGTGATGTTGT-3′; MAPK1-F: 5′-CGAAGCACCATTCAAGTTCGAC-3′; MAPK1-R: 5′-CTGAGCACGTCCAGTCCTCT-3′; PRKAR1A-F: 5′-GGGCCTTCTGATTATTTTGGTCAC-3′; PRKAR1A-R: 5′-CCCACAGGTTAGGGTCTCCT-3′; RAF1-F: 5′-GATGCCGTGTTTGATGGCTC-3′; RAF1-R: 5′-CCATTTCGCACATTGACCACT-3′; GAPDH-F: 5′-GGAGCGAGATCCCTCCAAAAT-3′; GAPDH-R: 5′-GGCTGTTGTCATACTTCTCATGG-3′. Calculation of fold change in gene expression was using the relative quantification (2− *ΔΔ*Ct) method.

### 2.10. Statistical Analysis

The values from cellular experiments are presented with mean ± standard deviation (SD) from three independently repeated experiments. Statistical analysis was calculated by IBM SPSS Statistics version 25.0 (SPSS Inc., Chicago, IL, USA) and GraphPad Prism version 8.0 (GraphPad Software, Inc., La Jolla, CA, USA). Differences between ischemia and control group were evaluated using Student's *t*-test. A one-sided *P* value <0.05 was deemed statistically significant.

## 3. Results

### 3.1. Workflow Diagram

Figure 1 shows the process of analysis for our work. The first step of our work was to identify 44 DEARGs from GSE61144 and HADb. Then, we did functional enrichment analysis, construction of PPI network, and key module analysis by Metascape. Next, DEmiRNAs were identified from GSE31568, and miRNAs and lncRNAs were predicted by multiple databases. LncRNA-miRNA-mRNA ceRNA regulation network was built, while hub genes were extracted. Subsequently, the immune cell composition and differences between AMI and normal groups were analyzed by CIBERSORT algorithm, and hub genes and immune cells were analyzed by Pearson correlation analysis. Finally, we verified the findings in this work through multidimensional aspects of another dataset and cellular experiments qPCR.

### 3.2. Identification of DEARGs in AMI Patients

In our work, 7 AMI and 10 normal samples from the dataset GSE61144 were analyzed, and 1645 DEmRNAs were identified, of which there were 904 upregulated and 741 downregulated (|logFC | >0.5 and adj. *P* value <0.05; Figure 2(a)). In parallel, 232 ARGs were obtained from HADb. Then, the 1645 DEmRNAs identified in GSE61144 were intersected with 232 ARGs. The outcome demonstrated that 44 DEARGs were used for the subsequent analysis (Figure 2(b)) and the gene expression was shown in the heat map (Figure 2(c)).

### 3.3. Functional Enrichment Analysis, PPI Network Construction, and Module Selection

To further screen genes associated with AMI onset and development, we made GO and enrichment analysis to access the biological functions of these 44 genes; at the same time, a PPI network was built to locate hub genes. The results of the functional enrichment analysis and PPI network by Metascape are shown in Figure 3.  Figure 3(a) shows that these DEARGs were majorly enriched in autophagy, apoptotic signaling pathway, response to starvation, apoptosis, and regulation of autophagy. To better understand the correlation between DEARGs and AMI, we analyzed the PPI network and MCODE components.  Figure 3(b) shows the network of enriched terms. Based on the results of MCODE component analysis (Figures 3(c)–3(e)), the biological functions of MCODE were found to be mainly related to PID ceramide pathway, corticotropin-releasing hormone signaling pathway, and autophagy, and we extracted the genes of MCODE from the PPI network for subsequent analysis.

### 3.4. Construction of miRNA-lncRNA-mRNA ceRNA Regulation Network

For the purpose of exploring the gene functions and regulatory mechanisms of DEARGs at a deeper level to understand the molecular mechanisms of AMI in a more in-depth and comprehensive manner, we constructed the ceRNA regulation network. We analyzed 20 AMI and 64 control samples from the dataset GSE31568, and 318 differentially expressed miRNAs (DEmiRNAs) were identified. As shown in Figure 4(a), there are 143 upregulated DEmiRNAs and 145 downregulated DEmiRNAs. 44 DEARGs were used to predict target miRNAs by Starbase, miRDB, and DIANA-TarBase v.8. We identified 285 mRNA-miRNA relationship pairs based on mRNA-miRNA interrelationships that were predicted simultaneously in all three databases. The 145 predicted miRNAs were compared with the 318 identified DEmiRNAs, and 47 miRNAs were extracted. We selected miRNA-mRNA relationship pairs with opposite expression to obtain 29 miRNAs. We then used Starbase, miRcode, and lncbase to predict the target lncRNAs using 29 miRNAs. And we identified 162 pairs of lncRNA-mRNA relationship pairs. After removing the miRNAs with no predicted results and the corresponding mRNAs, there were 45 lncRNAs, 24 miRNAs, 19 mRNAs, 162 lncRNA-miRNA pairs, and 37 mRNA-miRNA pairs.

We constructed ceRNA networks based on mRNA and miRNA expression profiles from AMI patients, and miRNAs and lncRNAs predicted by several databases, according to lncRNA-miRNA and miRNA-mRNA interactions (Figure 4(b)). These 19 mRNAs in the ceRNA network were intersected with 6 genes in MCODE of the PPI network, obtaining 4 autophagy-related hub genes, BCL2, MAPK1, RAF1, and PRKAR1A for subsequent analysis. Only these 4 genes were selected because they showed the greatest significance in the analysis results of DEARGs screening, PPI network construction, and ceRNA construction rather than other unregulated/downregulated DEARGs.

### 3.5. Analysis of Immune Cell Infiltration

In an attempt to uncover the association between the immune microenvironment and the development of AMI, we applied the CIBERSORT algorithm to evaluate the proportion of immunocytes from all samples in GSE61144.  Figure 5(a) shows a histogram of their relative composition for the 22 immune cell classes. CD8^+^ T cells, CD4^+^ T cells naive, NK cell resting, monocytes, and neutrophils were the major enriched immune cell subsets. The results of principal component analysis (PCA) showed significant group differences in immunocytes between AMI and controls (Figure 5(b)). Then, we compared the immunocyte composition of AMI and controls. The proportion of CD8^+^ T cells (*P* < 0.001), Tregs (*P* < 0.01), and mast cells resting (*P* < 0.05) were markedly less in AMI than normal group, whereas neutrophils (*P* < 0.001) and macrophages M0 (*P* < 0.001) were markedly greater than normal group (Figure 5(c)).

The correlation of 17 kinds of immunocytes was counted (since 5 kinds of immune cells were not estimated in all samples, they were not included in the correlation analysis) (Figure 5(d)). The heat map shows that the different subpopulations of immune cells show varying degrees of correlation. CD8^+^ T cells were markedly correlated with T cells gamma delta (*r* = 0.76, *P* < 0.01), NK cells resting (*r* = 0.61, *P* < 0.01), and mast cells resting (*r* = 0.54, *P* < 0.05) positively, yet markedly correlated with macrophages M0 (r = -0.58, *P* < 0.05) and neutrophils (*r* = −0.70, *P* < 0.01) negatively. Neutrophils were markedly correlated with CD4^+^ T cells memory activated (*r* = 0.67, *P* < 0.01) positively, but markedly correlated with CD8^+^ T cells (*r* = −0.70, *P* < 0.01), T cells regulatory (Tregs) (*r* = −0.70, *P* < 0.01), NK cells resting (*r* = −0.79, *P* < 0.01), and monocytes (*r* = −0.65, *P* < 0.01) negatively.

### 3.6. Co-Expression Analysis for DEARGs and AMI-Associated Immunocytes

The correlation between the 4 DEARGs and the 5 kinds of immune cells was analyzed further based on the findings of the previous analysis (Figure 6(a)). As shown in Figure 6(b), BCL2 is correlated with CD8^+^ T cells (*r* = 0.60, *P* < 0.05) positively, but correlated with neutrophils (*r* = −0.5, *P* < 0.05) negatively. MAPK1 was correlated with neutrophils (*r* = 0.75, *P* < 0.001) positively, but correlated with CD8^+^ T cells (*r* = −0.82, *P* < 0.001) negatively. PRKAR1A was correlated with neutrophils (*r* = 0.82, *P* < 0.001) positively, but correlated with CD8^+^ T cells (*r* = −0.76, *P* < 0.001) negatively. RAF1 was correlated with neutrophils (*r* = 0.88, *P* < 0.001) positively, but correlated with CD8^+^ T cells (*r* = −0.86, *P* < 0.001) negatively.

These findings indicate that DEARGs, which include BCL2, MAPK1, RAF1, and PRKAR1A, may have particular modulatory functions in immune infiltrating cells, specifically in CD8^+^ T cells and neutrophils.

### 3.7. Multidimensional Verification

Finally, we performed multidimensional validation in the dataset and cellular experiments qPCR, respectively. Validation is performed in 7 AMI (STEMI) and 7 control samples in the dataset GSE60993, and the results are shown in Figure 7(a). MAPK1 (*P* < 0.001), RAF1 (*P* < 0.001), and PRKAR1A (*P* < 0.05) were elevated in AMI, and conversely, BCL2 (*P* < 0.01) was decreased, which is congruous with our previous findings. We also performed cellular level experiments besides validation in the bioinformatics dataset. We cultured AC16 human cardiomyocytes in hypoxia for 4 hours and then ran qRT-PCR experiments to verify. The results are shown in Figure 7(b). MAPK1 (*P* < 0.05), PRKAR1A (*P* < 0.01), and RAF1 (*P* > 0.05) were elevated, and BCL2 (*P* < 0.05) was decreased in hypoxia cells compared with controls.

## 4. Discussion

Previous studies have searched and analyzed autophagy-related genes characterized in AMI patients. Bo's group identified functional variants of autophagy-related genes, for instance, ATG5 [40], ATG7 [41], ATG16L1 [42], and LC3B [43] in AMI patients. It has been identified that 7 DEARGs (WDFY3, TP53INP2, GABARAPL1, CDKN1A, DDIT3, NAMPT, and FOS) in AMI based on a feature selection algorithm, known as support vector machine-recursive feature elimination (SVM-RFE), which can be used to diagnose AMI as a potential biological marker [44]. On the other hand, it has been demonstrated in numerous studies that immune cells play an essential function in the development of AMI and postinfarction cardiac repair and remodeling [45, 46]. Previous work has found that there are N1 and N2 types of neutrophils in the myocardial infarction area. At an early stage post-MI period, proinflammatory type (N1) neutrophils showed a powerful proinflammatory and proinjury impact. The ratio of anti-inflammatory type (N2) was found to be increased over time and participated in the injury repair response after MI, exerting anti-inflammatory and anti-injury effects [47, 48]. Xia et al. found that Tregs were highly enriched in the myocardium of MI mice, and demonstrated that Sparc (secreted acidic cysteine-rich glycoprotein), which is highly expressed by cardiac Tregs, could protect the heart by increasing collagen content and enhancing maturation in the infarct scars to protect the heart [49]. For this research, we determined 4 autophagy-related genes (BCL2, MAPK1, RAF1, and PRKAR1A) associated with the occurrence of AMI. Besides, we found differences in 5 immune cell fractions (CD8^+^ T cells, Tregs, mast cells resting, macrophages M0, and neutrophils) by comparing the proportion of immunocytes between AMI and normal groups.

BCL2 can inhibit apoptosis in a variety of cell systems. Naseroleslami et al. found reduced BCL2 mRNA expression in an AMI rat model [50], which is consistent with our analysis. Ni et al. co-expressed BCL2 and vascular endothelial growth factor (VEGF) in mesenchymal stem cells (MSC), which could protect MSC by suppressing apoptosis, inhibiting autophagy and enhancing paracrine effects in an ischemic environment, and offering a new possibility for stem cell transplantation for the management of ischemic cardiac disease [51]. Kitabayashi et al. transplanted myoblast sheets overexpressing BCL2 into AMI rat model and effectively prolonged the survival time of myoblast sheets, reduced fibrosis in the myocardium, increased vascular density in the zones of infarction and margins, and improved cardiac function [52]. It has been observed in previous studies that neutrophils firstly infiltrate the infarcted area within a few hours after the onset of AMI, becoming abundant within 24 h, peaking on day 3, starting to fall back on day 5, and decreasing to lower levels until day 7, but still above baseline levels [45–48, 53]. Our research found that neutrophils were significantly elevated in patients within 4 h after the onset of AMI in agreement with the previous studies. However, BCL2 can inhibit neutrophil apoptosis [54]. It seems contradictory, but no relevant studies are available in AMI, and further exploration is needed. In summary, it appears that a new perspective may be offered for the treatment of AMI by intervening in BCL2.

MAPK1 encodes for one of the members of the MAP kinase family. MAP kinases, which are also named extracellular signal-regulated kinases (ERK), are participating in various cellular activities, for instance, proliferation, differentiation, transcriptional regulation, and development. Zhou et al. observed that MAPK1 was elevated in the MI/RI mice model and isoflurane could improve hemodynamics and myocardial injury by upregulating miR-378 to inhibit MAPK1 [55]. This was compatible with our results. Ruan et al. found that knockdown of lncRNA DANCR could attenuate cardiomyocyte injury through miR-19a-3p/MAPK1 axis [56]. Yu et al. found CD8^+^ T cells decreased on day one in AMI patients by bioinformatic analysis [57] in line with our results. D'Souza et al. found that Erk2 (MAPK1) can affect CD8^+^ T cells via cell activation, proliferation, and survival aspects and is crucial for the survival of activated CD8^+^ T cells in vivo [58].

RAF1 is involved in activating the MAPK cascade reactions. Jiang et al. detected upregulated RAF1 and MAPK1 in extracellular vesicles (EV) in the plasma of AMI patients at 4-6 hours after onset, which is consistent with our findings [59]. Zhang et al. found that RAF1 was consistently upregulated from day 7 to day 28 after MI in neonatal pigs [60]. Cai et al. showed that activation of RAF1 through downregulation of miR-146b-3p contributes to the activation of the RAF/P38MAPK/COX-2 signaling pathway, which in close relation with the progression of diabetic brain infarction [61]. MAPK signaling is crucial for T cell development [62], activation [63], proliferation, and survival [58]. Several selective inhibitors of ERK signaling, such as FR180204, BVD523, CC90003, GDC-0994, MK-8353, and BVD523 (ulixertinib), have been reported to have significant antitumor efficacy, but more exploration is needed because MAPK inhibition may lead to T cell depletion and/or unresponsiveness in some cases due to the important role of MAPK in T cell function [64]. Given the efficacy achieved in tumor therapy and the preliminary work in AMI, intervening in genes such as MAPK1 and RAF1 and modulating the MAPK cascade response may lead to new therapeutic options for AMI.

PRKAR1A is a protein-encoding gene that encodes protein kinase A (PKA) regulatory subunit 1*α* (R1*α*). PKA is a critical modulator of cardiac contractility and heart rate [65], and its dynamic regulation is essential for cardiac homeostasis. It was demonstrated that abnormal activation or deactivation of PKA is strongly associated with the progression of cardiovascular diseases, for instance, myocardial ischemia, hypertrophy, and heart failure [65]. R1*α* is expressed at a high level in the heart and regulates PKA activity by chelating PKA catalytic subunits [66]. Zhang et al. found that when cardiac contractility is reduced, decreased PKA activity/activation leads to a reduction in cardiac reserve and exercise capability [67]. Liu et al. identified PRKAR1A as a highly scored necrosis suppressor gene by a genome-wide RNAi screen [68]. This team then subsequently found that unrestricted PKA activation induced by R1*α* deficiency exacerbates oxidative stress, myocardial cell necrosis, and myocardial I/R injury [69]. PRKAR1A has been less studied in AMI. Our results showed different results from Liu's, probably related to cell type and modeling methods. However, our and Liu's views are in agreement with previous work that abnormal activation or inactivation of PKA contributes to myocardial ischemic injury. Taken together, PKA may be a hopeful pharmacological target for improving clinical outcomes and protecting the heart after MI.

The current treatment of AMI mainly consists of drug therapy and reperfusion therapy [1, 2]. Despite the great advances in the treatment of myocardial infarction in recent decades, the efficacy and safety of new therapies for myocardial repair or prevention of adverse remodeling (e.g., cell therapy or gene therapy) have not been achieved [2]. There is an urgent need for new therapeutic approaches to improve the treatment. Fortunately, it has been found that some drugs can target DEARGs or autophagic mechanisms to treat the disease. For example, in other subject areas, Alhoshani et al. found that venetoclax (BCL2 inhibitor) could suppress the cell growth and proliferation of triple-negative breast carcinoma by inducing autophagy-associated cell apoptosis and cycle arrest, as well as death [70]. Zhang et al. designed LYN-1604, an agonist of the autophagy gene ULK1, which can induce ATG5-dependent autophagic death in triple-negative breast carcinoma cells by activating the ULK complex [71]. Jiang et al. found that the SGLT2 inhibitor empagliflozin (EMPA) could exert cardioprotective effects by downregulating autophagic flux in vivo and in vitro models of MI [72]. There have been several studies on the regulation of autophagy-related genes in immune cells. Lagasse et al. found that BCL2 inhibited neutrophil apoptosis in BCL2-overexpressing transgenic mice [54]. D'Souza et al. found that Erk2 (MAPK1) can affect CD8^+^ T cells in multiple ways, including cell activation, proliferation, and survival, and is required for the survival of activated CD8^+^ T cells in vivo [58]. Besides the autophagy-related genes and immune cells involved in our study, ATG5 has been found to regulate host innate and adaptive immune responses by regulating dendritic cell activation [73]. Since autophagy can affect the proliferation, differentiation, survival, and apoptosis of immune cells and is also regulated by various cytokines, studying the mechanisms of communication and regulation between autophagy and immune cells in AMI will not only help to further investigate the disease mechanism of AMI, but also may be a new direction and therapeutic target for the treatment of AMI.

Autophagy is a fundamental cellular metabolic process, an autonomous degradation modality that is involved in the formation and progression of AMI with a two-sided character [12], while possibly interacting with various immune cells that together complete the complex process of AMI development. In conclusion, we hypothesize that DEARGs may have an impact in the progression of AMI through influencing immune cells to modulate the inflammatory response. Previous reports have shown that cellular autophagy or immunocytes are strongly associated with the progression of AMI. However, there has been no systematic study to elucidate the association of autophagy genes with immune cells in AMI patients. So far as we know, here is the first research systematic integrated study of autophagy-related genes and immune infiltrating cells in AMI patients.

Our study has some limitations that should be acknowledged as inevitable. The study was retrospective and could not access important clinical information, as well as the sample size was small; therefore, a greater sample size of a prospective study should be conducted to validate our conclusions. The present study inferred the potential mechanisms of 4 genes and 2 immune cells for the development of AMI by bioinformatics analysis, and further molecular mechanisms are needed to explore the potential associations and functions of cellular autophagy and immune infiltration in AMI patients.

## 5. Conclusions

We explored and analyzed DEARGs and the distribution of immune cells in AMI by bioinformatics and qPCR experiments and constructed a miRNA-lncRNA-mRNA ceRNA network. Ultimately, we identified 4 autophagy-related hub genes, BCL2, MAPK1, RAF1, and PRKAR1A, that may play particular modulatory effects in immune infiltrating cells, notably in CD8^+^ T cells and neutrophils. This work not only contributes to new findings on the mechanisms of autophagy and immune regulation in AMI, but also may provide potential diagnostic markers and new perspectives for the treatment of AMI.

## Figures and Tables

**Figure 1:** The flowchart of the analysis process.

**Figure 2:** Identification of differentially expressed autophagy-related genes in AMI patients. (a) Volcano plot of differentially expressed genes between the two groups of samples in GSE61144. The red points represent upregulated genes screened on the basis of logFC > 0.5 with an adj. *P* value <0.05. The green points represent downregulated genes screened on the basis of logFC < −0.5 with an adj. *P* value <0.05. The black dots represent genes with no significant difference. FC is the fold change. (b) Venn diagram of the intersection of DEmRNAs and ARGs in HADb. The dark area in the middle represents DEARGs that were identified by analysis of DEmRNAs (left, purple) and ARGs in the Human Autophagy Database (HADb) (right, orange). (c) Heat map of DEARGs. Red indicates that gene expression is relatively upregulated, green indicates gene expression is relatively downregulated, and black indicates no significant change in gene expression.

**Figure 3:** The enrichment analysis of 44 DEARGs in AMI (Metascape). (a) Bar graph of top 20 enriched terms across DEARGs, colored by *P* values. (b) Network of enriched terms, colored by cluster ID. (c, d, and e) Protein-protein interaction network and MCODE components identified in DEARGs.

**Figure 4:** Volcano plot of miRNAs and ceRNA network. (a) Volcano plot of differentially expressed data between the two groups of samples in GSE31568. The red points represent upregulated miRNAs screened on the basis of logFC > 0.5 with an adj. *P* value <0.05. The green points represent downregulated miRNAs screened on the basis of logFC < −0.5 with an adj. *P* value <0.05. The black dots represent genes with no significant difference. FC is the fold change. (b) View of miRNA-lncRNA-mRNA ceRNA regulation network, and the ellipse, rectangle, and diamond represented mRNA, miRNA, and lncRNA, respectively.

**Figure 5:** Analysis of immune cell infiltration in AMI and controls of GSE61144. (a) Bar plot showing the relative fraction of 22 immune cell clusters in all samples. (b) Principal component analysis (PCA) was performed on all samples. Principal components 1 and 2 accounted for 93.8% of the total components. Orange represents the normal group and green represents the STEMI group. (c) The box plot comparing the immune cell composition of the STEMI and normal groups. Orange represents the normal group and green represents the STEMI group. ^∗^ represents *P* < 0.05, ^∗∗^ represents *P* < 0.01, ^∗∗∗^ represents *P* < 0.001. (d) Pearson correlation analysis of different immune cell subsets.

**Figure 6:** Co-expression analysis for DEARGs and AMI-associated immunocytes. (a) Pearson correlation analysis of 4 DEARGs (BCL2, MAPK1, RAF1, and PRKAR1A) and 5 immune cells (CD8^+^ T cells, Tregs, mast cells resting, macrophages M0, and neutrophils). (b) Scatter plot of the relationship between hub DEARGs (BCL2, MAPK1, RAF1, and PRKAR1A) and immune cells (CD8^+^ T cells and neutrophils), respectively. *R* and *P* values are labeled on the images.

**Figure 7:** Validation by dataset and qPCR. (a) In the dataset GSE60993, we analyzed 7 STEMI and 7 normal samples and showed that MAPK1, RAF1, and PRKAR1A were elevated in STEMI, and conversely, BCL2 was decreased. (b) The relative expression levels of the 4 DEARGs were detected by qPCR in AC16 cells. The data are expressed as the mean ± standard error of measurement from at least three experiments. ^∗^ represents *P* < 0.05, ^∗∗^ represents *P* < 0.01, ^∗∗∗^ represents *P* < 0.001.

## Data Availability

These data were derived from the following resources available in the public domain: GSE61144 (https://www.ncbi.nlm.nih.gov/geo/query/acc.cgi?acc=gse61144), GSE31568 (https://www.ncbi.nlm.nih.gov/geo/query/acc.cgi?acc=GSE31568), and GSE60993 (https://www.ncbi.nlm.nih.gov/geo/query/acc.cgi?acc=GSE60993).

## Abbreviations

AMI: Acute myocardial infarction
CHD: Coronary heart disease
DEARGs: Differentially expressed autophagy-related genes
PPI: Protein-protein interaction
CIBERSORT: Cell type identification by estimating relative subsets of RNA transcripts algorithm
I/R: Transcripts algorithm
GEO: Gene Expression Omnibus
FC: Fold change
STEMI: ST elevated myocardial infarction
DEmRNAs: Differentially expressed mRNAs
DEmiRNAs: Differentially expressed miRNAs
HADb: The human autophagy database
GO: Gene ontology
KEGG: Kyoto Encyclopedia of Genes and Genomes
ARGs: Autophagy-related genes
PCA: Principal component analysis
Tregs: Regulatory T cells.
